# 3D Virtual Reality Implementation of Tourist Attractions Based on the Deep Belief Neural Network

**DOI:** 10.1155/2021/9004797

**Published:** 2021-09-11

**Authors:** Fuli Song

**Affiliations:** Academy of Design Arts, Xijing University, Xi'an 710123, Shannxi, China

## Abstract

In today's society, information technology is widely used, and virtual reality technology, as one of the emerging frontier technologies, has entered a stage of rapid development. Virtual reality is the use of computer technology to simulate the real-life environment into a virtual simulation environment, with the help of special equipment to realize the natural interaction between users and technical environment, in which the tourism industry is the most widely used. In order to realize 3D virtual reality of tourist attractions and improve users' immersive experience in the process of interaction, the deep belief neural network is introduced to realize the target recognition and reconstruction in virtual reality. The results show that the algorithm has excellent performance in target recognition and target reconstruction, and deep belief networks improve the accuracy by 0.57% and 0.81% and the accuracy by 0.21% and 2.06%, respectively, compared with the current optimal algorithm in target recognition of 12 and 20 view regular projection images. Compared with the current optimal algorithm, deep belief networks are reduced by 0.2%, 3.7%, and 0.6%, respectively. The accuracy index was increased by 2%, 0.1%, and 0.1%, respectively. The above results show that the proposed algorithm based on the deep belief neural network can realize 3D virtual reality of complex scenes such as tourist attractions according to its excellent performance.

## 1. Introduction

Nowadays, the continuous breakthrough of information technology has brought great impact on people's production and life. The rapid development of virtual reality technology provides a new idea for the transformation and development of traditional tourism form. Using this technology can give tourists an immersive and unique virtual reality experience. This is an emerging technology integrating intelligent pattern recognition, computer graphics, machine vision, and other disciplines [1]. Tourists can get an immersive experience interacting with the simulation environment without leaving home. However, in practical application, especially in the realization of 3D virtual reality of tourist attractions, there are three technical difficulties in complex scenes, including target recognition, target reconstruction, image display, and human-computer interaction [2]. Among them, target recognition and target reconstruction are the keys to the realization of virtual reality. When target recognition is carried out in tourist attractions, there will be many kinds of targets, easy occlusion, complex texture background, large gap in volume, and shape. Traditional recognition methods are easy to lose key information and reduce the accuracy of target detection. When reconstructing the target, the traditional structure from motion (SFM) [3] has poor robustness and adaptability, which will reduce the reconstruction accuracy of the target and directly affect the quality of user experience. These also become the problems to be solved to improve the virtual reality implementation technology and user experience. In order to further understand the above problems, we refer to the research of the LSTM neural network algorithm based on particle swarm optimization in anomaly detection and the technology of sensor data and recursive network in 3D virtual reality. The conclusion is that the current deep confidence neural network algorithm can effectively solve this kind of problem.

With the rapid development of the deep belief neural network, the shortcomings of traditional algorithms such as SFM become increasingly prominent, such as the large amount of calculation, and the traditional algorithms can only select the artificial features when extracting the image features, which leads to some important information missing and affects the effect of image reconstruction. Therefore, many scholars begin to focus on the deep neural network. Ma et al. first proposed the idea of using encoding and decoding to construct the mapping relationship between two-dimensional image and three-dimensional image through the deep neural network and extracted two-dimensional model feature vectors from the traditional convolutional neural network through deconvolution network decoding to reconstruct the three-dimensional model [4]. Lu et al. proposed a 3D recurrent neural network framework 3D-R2N2 (3D recurrent reconstruction neural network) based on the deep neural network and reconstructed the 3D model by estimating the pixel probability density [5]. Peng et al. proposed a graph-based depth belief neural network GCN (graph neural network), which can reconstruct the 3D model of a single RGB image [6]. Hu et al. proposed the first deep neural network framework PointNet to directly process point cloud, which realized the tasks of classification and recognition and semantic segmentation of point cloud data objects [7]. Later, Lin et al. proposed PointNet + neural network architecture [8] for the problems of PointNet in dealing with local features. Based on the convolution operation directly used on the point cloud, Hu et al. constructed a point cloud network for 3D semantic segmentation and target recognition tasks [9]. Wang et al. used a three-dimensional convolutional depth belief network (DBN) to recognize targets and predict viewing angles with three-dimensional voxels as inputs [10]. The network LightNet designed by Hou et al. is lightweight and has higher recognition performance and efficiency [11]. Wang et al. used the advantages of octree to store 3D voxel data and proposed a convolutional neural network O-CNN (octree-based convolutional neural networks) with high training speed [12]. Wang et al. proposed the MVCNN (multiview convolutional neural networks) to obtain a series of two-dimensional rendering images of three-dimensional objects by the multiview projection method and then obtained the three-dimensional object shape feature description of the image through feature extraction for recognition and classification [13]. Based on the MVCNN framework, Deng et al. proposed the cyclic clustering pooling operation. By adding feature information, the MVCNN perspective pooling was extended to multilevel pooling, and the original framework was improved, which achieved good results in practical application [14]. Chen et al. proposed the FusionNet network framework with three neural networks and obtained a more complete representation of 3D target features [15].

To sum up, many scholars have carried out a lot of research on the neural network, virtual reality, target recognition, target reconstruction, and so on [16–22]. Traditional algorithms such as SFM, which are used to realize 3D virtual reality of tourist attractions, are prone to information loss, feature omission, and low accuracy in target recognition and reconstruction; due to their large amount of calculation and poor adaptability, it directly affects tourists' 3D virtual reality experience in tourist attractions. In view of this, the deep belief neural network is introduced, which can obtain a complete two-dimensional projection image from the three-dimensional scene and realize the target recognition and reconstruction, so as to better realize the 3D virtual reality of tourist attractions.

## 2. Virtual Reality Implementation of Tourist Attractions Based on the Deep Belief Neural Network

### 2.1. Scenic Spot Target Recognition Based on the Depth Belief Neural Network

Aiming at the 3D target recognition task of multiview of tourist attractions, a multiview feature fusion strategy based on the depth belief neural network is proposed. The diagram is shown in Figure 1. The method is composed of three modules: two-dimensional convolutional neural network (CNN), multilayer residual LSTM subnetwork [23], and multiview feature weighted fusion. The convolutional neural network (CNN) module is responsible for image feature extraction. Compared with the traditional artificial feature extraction, this module can enhance the image feature and reduce the influence of noise; The multilayer residual LSTM subnetwork can obtain the association information between multiple images of different views of the 3D model, so as to analyze the correlation of image features of each model sequence. Finally, the multiview feature weighted fusion module can perform feature weighted fusion for each associated view to further improve the recognition ability of the algorithm.

The first step is the CNN convolution feature extraction. ResNet18 is selected as a two-dimensional neural network for low-level feature extraction. Convolution feature extraction is performed on the original input multiview regular projection image to obtain a series of low-level feature description vectors [24]. ResNet18 means that the neural network is mainly composed of 17 convolution layers and 1 full connection layer, and the network depth is 18. Its network architecture is shown in Figure 2. In the graph, the solid line jump represents the new feature vector generated by the addition of two feature graphs, and the dotted line jump represents that the convolution operation is needed to make the high and low convolution features consistent before the feature addition. Through the feature extraction of this method, we can optimize the network structure, deepen the network depth, and improve the recognition accuracy. The convolution features obtained by the network are used as the input of the extraction network. For the CNN, not all the upper and lower neural units can be directly connected, but through the “convolution kernel” as the intermediary, the same convolution kernel can be directly connected and used in most images. Finally, the extracted feature points still maintain their original position and are connected to the LSTM layer. The LSTM network layer prevents the gradient from disappearing through its own time memory function and obtains the characteristic points transmitted by the CNN layer for training operation.

The network layer in Figure 2 represents only the convolution layer and the full connection layer depth architecture.

The second step is to extract the sequence features of the multilayer RES-LSTM subnetwork. The multiview feature map obtained in the first step is taken as the feature map of the recurrent neural network LSTM to obtain the correlation features among the views. LSTM is a special variant of the neural network, which has a repetitive network module. The difference between the LSTM and ordinary recurrent neural network is that it solves the long-term dependence problem of long sequence data information by introducing gating unit. The unit structure is shown in Figure 3, which is composed of memory unit, input gate, output gate, and forgetting gate. Each part corresponds to the operation process of LSTM unit, and the specific update formula can be expressed as follows:

(1) $$\begin{array}{c} \left\{\begin{array}{c} i_{t}=\sigma \left(W_{i}x_{t}+U_{i}h_{t-1}+b_{i}\right),\\ o_{t}=\sigma \left(W_{\text{o}}x_{t}+U_{\text{o}}h_{t-1}+b_{\text{o}}\right),\\ f_{t}=\sigma \left(W_{f}x_{t}+U_{f}h_{t-1}+b_{f}\right),\\ {\tilde{c}}_{t}=\tanh\left(W_{c}x_{t}+U_{c}h_{t-1}+b_{c}\right),\\ c_{t}=i_{t}⊙{\tilde{c}}_{t}+f_{t}⊙c_{t-1},\\ h_{t}=o_{t}⊙\;\tanh\left(c_{t}\right). \end{array}\right) \end{array}$$

In formula (1), *f*_*t*_, *i*_*t*_, and *o*_*t*_ represent the forgetting gate, input gate, and output gate in turn, ${\tilde{c}}_{t}$ represents the candidate information obtained from input *x*_*t*_ at the current time and hidden state *h*_*t*−1_ at the previous time, and *c*_*t*_ represents the internal state of memory unit.

LSTM unit achieves the fusion of sequence information through its own special mechanism and obtains the association information between the sequence images to obtain the complete data information of 3D target. In order to further improve the accurate recognition performance of 3D targets, a 5-layer RES-LSTM network is constructed based on the residual idea, and its structure is shown in Figure 3.

As can be seen from Figure 3, the LSTM network realizes sequence information fusion such as the CNN network layer through its own memory mechanism. The feature correlation points between the sequence images are obtained to form the specific data of the three-dimensional target. The third step is the weighted fusion of multiview features, which is the weighted fusion of the association features among the views in the second step to obtain a more advanced feature combination vector to improve the recognition performance of the model. According to the mechanism of LSTM unit, the hidden state *h*_*t*_ output at each time has part of the effective information of the previous time, that is, the hidden state *h*_*n*_ at the last time has the most effective information. Therefore, the subcontributions of the hidden state *h*_*t*_ to the object shape description at each time are different, and with the increase of the input sequence time, the more information it retains. The weight contribution of the description of the target shape is higher. Its structure is shown in Figure 4. The variable of *X* is defined to represent the target morphological feature points of each scene. With the increase of time series, the final identified target is obtained after the LSTM network hidden state analysis.

In order to recognize the shape of the target accurately, a multiview feature fusion strategy is proposed:

(2) $$\begin{array}{c} H=\sum_{i}^{N}\omega_{i}h_{i}. \end{array}$$

In equation (2), *H* is the descriptor of the final 3D target feature vector, *h*_*i*_ is the hidden state at each time, *ω*_*i*_ is the weight coefficient corresponding to different hidden states, and the weight coefficient is defined as

(3) $$\begin{array}{c} \omega_{i}=\frac{e^{ki}-e^{-ki}}{e^{ki}+e^{-ki}} \end{array}$$

Through the optimization experiment, when K in equation (3) is 0.4, the recognition accuracy of the model is the highest.

### 2.2. Scenic Spot Target Reconstruction Based on the Depth Belief Neural Network

For the reconstruction of 3D objects in tourist attractions, the traditional SFM algorithm is prone to the loss of part of the target information, resulting in the reconstruction of the surface of the target holes, large position deviation, and other problems. Therefore, a multiscale feature fusion strategy based on the deep belief neural network is proposed. The depth information of the corresponding image is predicted through the depth estimation of the two-dimensional RGB image, so as to reduce the depth prediction error of the SFM algorithm and improve the accuracy of the scenic spot target reconstruction. The strategy consists of three steps: feature extraction, multiscale fusion, and upsampling optimization. The actual intention is shown in Figure 5. First, the basic feature extraction network extracts low-level feature vectors sufficient to support subsequent modeling from the input two-dimensional image through the convolution neural network. Then, the multiscale feature fusion neural network fuses the low-level feature vectors to obtain the spatial structure information of the enhanced features. Finally, the depth estimation value of each pixel is obtained by the upsampling optimization network to obtain the depth estimation map of the target image. Complete the reconstruction of the goal.

The first step is to extract image features. Due to the stacking structure and convolution characteristics of the convolution neural network, feature vectors of different scales will be obtained after convolution operation. Multiple convolution operations will not only obtain features of different levels but also enrich the semantic information contained in features [25]. Therefore, DenseNet121 is selected as the basic feature extraction network of the multiscale feature fusion network, and its feature extraction diagram is shown in Figure 6. DenseNet121 is a dense convolutional neural network composed of 120 convolutional layers and one fully connected layer. The network depth is 121. It includes four dense connected network blocks, and each network block contains two convolutional layers. With the transmission of information in the network, feature maps of different scales are obtained.

The second step is the fusion of multiscale features to obtain the spatial structure information of enhanced features. The common method of multiscale feature extraction is to extract different scale feature images by DenseNet121 network feature extraction, scale the feature images to build image pyramids with different resolutions, and then extract the features of all resolution images by the convolution neural network, but a lot of memory is occupied in the calculation process The low operation speed limits the method greatly. The feature pyramid network (FPN) can obtain feature images of different sizes after multiple convolution and pooling operations on the original image according to its own characteristics of the convolution network, which is a top-down path to complete the fusion of different features [26]. In view of this, a multiscale feature fusion network for depth information estimation is proposed. The network structure is shown in Figure 7.

As can be seen from Figure 7, the operation process of the whole multiscale feature fusion network structure can be divided into three steps. First, the forward propagation of the basic network module “from bottom to top,” then the “top-down” and horizontal connection, and finally the deconvolution and feature fusion. By means of two-step fusion, the network not only preserves the details of image features but also has good feature resolution, which is more suitable for depth estimation of two-dimensional image.

The third step is to optimize the feature after multiscale feature fusion. The size of the feature image obtained by the multiscale feature fusion module is different, and it needs to be restored to the same size as the original image. The common method of image upsampling is to insert new elements by linear interpolation. Traditional linear interpolation algorithms include the bilinear interpolation method, nearest neighbor interpolation method, bicubic interpolation method, and so on [27–29]. In the process of up sampling, the traditional method is easy to cause mosaic and sawtooth phenomenon in the image, so the improved deconvolution method is used to avoid the above problems [30]. The specific operation is to first pool the uppooling layer, fill in the places lacking eigenvalues with zeros, and convolute all the places with zeros to get a new scale feature map. At the same time, in the case of the same scale, the residual idea and small convolution kernel are used to reduce the network parameters and improve the operation efficiency. Its structure is shown in Figure 8.

In depth image estimation of scenic spot target, depth estimation is usually regarded as a regression problem because the distance between the scenic spot target and sampling camera is continuous. The loss functions commonly used to solve regression problems include square loss, absolute value loss, Huber loss, and BerHu loss; among them, BerHu loss function has good robustness in processing monocular depth map estimation task, so we choose BerHu loss function as the training loss function of the network, and its formula is as follows.

(4) $$\begin{array}{c} \text{BerHu}=\left\{\begin{array}{cc} \left|x_{i}\right|, & \left|x_{i}\right|<c,\\ \frac{x_{i}^{2}+c^{2}}{2c}, & \left|x_{i}\right|\geq c. \end{array}\right) \end{array}$$

In equation (4), *x*_*i*_=*d*_*i*_^pre^ − *d*_*i*_^gt^, where *d*_*i*_^pre^ is the predicted depth value and *d*_*i*_^gt^ is the true value of the depth map. *C* is the threshold, and the specific value is 0.2max_1≤*i*≤*n*_|*d*_*i*_^pre^ − *d*_*i*_^gt^|, which is 0.2 times of the maximum residual of the whole image. Because the loss of initial depth map and refined depth map need to be considered at the same time, the BerHu loss of real depth map and estimated depth map is selected as the monitoring loss of training:

(5) $$\begin{array}{c} \text{Loss}=\sum \left(L_{p}+\lambda L_{r}\right). \end{array}$$

In equation (5), *L*_*p*_ is the BerHu loss of the initial depth map, *L*_*r*_ is the BerHu loss of the optimized depth map, and *λ* is taken as 1. Finally, it is summarized that the deep neural network receives information and transmits it to each company layer through the multipath unit neural network and responds by activation or inhibition. The calculated cell neural value is the input of data, and the reaction content is the network node. According to the depth data map of the real content, the loss degree of training is calculated to solve the regression problem.

## 3. Analysis of the Virtual Reality Effect of Tourist Attractions Based on the Deep Confidence Neural Network

### 3.1. Performance Comparison and Analysis of Virtual Reality Target Recognition for Scenic Spots

In order to verify the performance of virtual reality target recognition of tourist attractions, the multiview feature fusion strategy based on the deep belief neural network is evaluated and tested. The model net benchmark dataset commonly used for 3D target recognition is selected as the test dataset, which contains two different subsets of ModelNet10 and ModelNet40. The former contains 10 class targets and 4899 CAD models, while the latter contains 40 class targets and 12311 CAD models, and all of them are subject to angle artificial attitude alignment [31]. Generally speaking, the higher the accuracy, the better the overall classification effect of the recognition model. The higher the accuracy, the lower the false detection rate of the recognition model.

The model recognition accuracy is the total number of correct classification times divided by the number of all classification samples:

(6) $$\begin{array}{c} \text{Accuracy}=\frac{\text{TP}+\text{TN}}{\text{TP}+\text{TN}+\text{FP}+\text{FN}}. \end{array}$$

In equation (6), TP is the number of correct identifications, TN is the number of correct identifications of nonclass, FP is the number of wrong identifications of nonclass, and FN is the number of wrong identifications.

The accuracy rate is the proportion of the positive samples in the recognition algorithm. The calculation formula is as follows:

(7) $$\begin{array}{c} \text{Precision}=\frac{1}{n}\overset{n}{\underset{i=1}{\sum }}\frac{\text{TP}}{\left(\text{TP}+\text{FP}\right)}. \end{array}$$

In equation (7), *n* is the total number of categories, and *i* is the label of each category.

Then, the multiview feature fusion algorithm DBN based on the deep belief neural network is compared with the mainstream target recognition network algorithms of the MVCNN, MVCNN-New [32], and MVCNN-MultiRes [33] in 12 and 20 view regular projection images. The test results are shown in Figure 9 and Figure 10.

Figure 9 shows the test results of recognition performance of each algorithm in 12 regular projection images. The test results show that the DBN is superior to other algorithms in recognition accuracy. Compared with the second MVCNN-New, the accuracy and precision of the MVCNN-New are 95% and 92.4%, respectively. The accuracy and accuracy of the DBN are improved by 0.57% and 0.21% respectively.

Figure 10 shows the test results of recognition performance of each algorithm in 20 regular projection images. The test results show that the recognition accuracy of the DBN is significantly better than other algorithms. Compared with the second MVCNN-New, the accuracy and precision rate is 96.03% and 93.4%, and the accuracy and precision rate of the DBN is improved by 0.81% and 2.06%, respectively. It can be seen from the comparison results in Figures 9 and 10 that among various branches of the multiview feature fusion algorithm of the deep confidence neural network, the proposed model is obviously superior to other algorithms in recognition accuracy. It improves the recognition accuracy of projected images and is more suitable to participate in the research of 3D virtual reality technology of scenic spots.

### 3.2. Performance Comparison and Analysis of Virtual Reality Target Reconstruction in Scenic Spots

In order to verify the reconstruction performance of virtual reality target in tourist attractions, the multiscale feature fusion strategy based on the deep belief neural network is evaluated and tested. The NYU depth indoor depth map dataset published by New York University is selected as the test dataset, which includes NYU depth V1 and NYU depth V2. The former contains 7 different scene types and 64 different indoor scenes, and the latter contains 400000 scene RGB images and corresponding depth maps [34]. In order to facilitate the research and training, 1449 pieces are with the size of 640 × 480, with the corresponding annotation complete depth map and crisp chicken in a label of the accurate annotation image, as shown in Figure 11. 795 images were randomly divided into training data and 654 images as test data.

When evaluating the neural network algorithm of scenic spot target reconstruction, the evaluation index [35] of Laina et al.' model is generally selected, which includes the following six aspects.

The root mean squared error (RMSE) is expressed as

(8) $$\begin{array}{c} \text{RMSE}=\frac{1}{T}\overset{T}{\underset{i=1}{\sum }}{\left(d_{i}^{\text{gt}}-d_{i}\right)}^{2}. \end{array}$$

The average relative error (REL) is expressed as

(9) $$\begin{array}{c} \text{REL}=\frac{1}{T}\overset{T}{\underset{i=1}{\sum }}\frac{\left|d_{i}^{\text{gt}}-d_{i}\right|}{d_{i}^{\text{gt}}}. \end{array}$$

The average log10 error (log10) formula is expressed as

(10) $$\begin{array}{c} \log_{10}=\frac{1}{T}\overset{T}{\underset{i=1}{\sum }}\left|\log_{10}d_{i}^{\text{gt}}-\;\log_{10}d_{i}\right|. \end{array}$$

The accuracy rate under the three thresholds is *δ*:

(11) $$\begin{array}{c} \delta_{i}=\max\left(\frac{d_{i}^{\text{gt}}}{d_{i}},\frac{d_{i}}{d_{i}^{\text{gt}}}\right)<1.25^{i}\;\left(i=1,2,3\right), \end{array}$$

where *d*_*i*_^gt^ is the true depth value, *d_i_* is the estimated depth value, and *t* is the total number of pixels. The lower the values of RMSE, REL, and log10, the higher the reconstruction accuracy of the algorithm model, while the three accuracy indexes *δ* are on the contrary.

Ablation experiment of the multiscale feature fusion module in the network under the condition of monocular depth estimation is using the NYU depth V2 dataset. As can be seen from Figure 12, the performance of the multiscale feature fusion module is further improved compared with the direct use of convolution feature map for depth map prediction.

Figure 13 shows the ablation experiment on the feature fusion module of the upsampling optimization module in the network under the condition of monocular depth estimation using the NYU depth V2 dataset. It can be seen from Figure 13 that the upsampling optimization module optimizes the original RGB image and the initial depth map obtained by deconvolution. Compared with the initial depth map obtained by deconvolution directly, its performance evaluation indexes are further improved, and the structure details of the depth map are clearer.

Figure 14 shows the performance test of the mainstream depth estimation algorithms, such as the Eigen [36], Laina [35], and DBN, on the reconstruction of scenic spots using the NYU depth V2 dataset. The results show that the DBN is superior to other algorithms in target reconstruction accuracy. Compared with the current optimal Laina algorithm model, the DBN algorithm reduces REL by 0.2%, RMSE by 3.7%, and log10 by 0.6% and improves accuracy by 2%, 0.1%, and 0.1%, respectively. Using this algorithm to deal with the complex environment and rich scene information of tourist attractions, we can obtain more precise depth information and provide more accurate target reconstruction image in the realization of 3D virtual reality of tourist attractions.

## 4. Conclusion

The application and development of virtual reality technology in tourism industry is a typical representative of the popularization of information technology. In this study, a feature fusion scheme based on the deep belief neural network is proposed to solve the problems of information loss, feature omission, and low accuracy in the process of 3D virtual reality of tourist attractions. The unsupervised learning characteristics of the deep belief neural network are used to retain the original features as much as possible. It can improve the accuracy of recognition and reconstruction in the realization of virtual reality. The scheme can retain more details for the 3D virtual reality implementation of tourist attractions and bring tourists a better immersive experience. The results show that the algorithm has excellent performance in target recognition and target reconstruction, and deep belief network improves the accuracy by 0.57% and 0.81% and the accuracy by 0.21% and 2.06%, respectively, compared with the current optimal algorithm in target recognition of 12 and 20 view regular projection images. Compared with the current optimal algorithm, deep belief networks are reduced by 0.2%, 3.7%, and 0.6%, respectively. The accuracy index *δ* < 1.25^1^, *δ* < 1.25^2^, *δ* < 1.25^3^ was increased by 2%, 0.1%, and 0.1%, respectively. The above results show that the new algorithm has better adaptability and higher accuracy in the realization of 3D virtual reality in complex environments such as tourist attractions and can greatly reduce the problems of missing information, missing features, and low accuracy in target recognition and reconstruction. This research combines the deep belief network with virtual technology, which provides a new exploration direction for the realization of 3D virtual reality in tourist attractions.

## Figures and Tables

**Figure 1:** Schematic diagram of target recognition based on the DBN.

**Figure 2:** ResNet18 network model diagram.

**Figure 3:** LSTM internal structure and multilayer RES-LSTM module.

**Figure 4:** Schematic diagram of multiview fusion feature structure.

**Figure 5:** Schematic diagram of target reconstruction based on the DBN.

**Figure 6:** Schematic diagram of feature extraction for DenseNet121 network structure.

**Figure 7:** Design of the multiscale feature fusion module.

**Figure 8:** Structure diagram of the upsampling module.

**Figure 9:** Comparison and evaluation results of each algorithm on the ModelNet dataset from 12 views.

**Figure 10:** Comparison and evaluation results of each algorithm on the ModelNet dataset from 20 views.

**Figure 11:** Examples of RGB images, original depth images, and class labels in the NYU depth dataset.

**Figure 12:** Experimental results of the multiscale fusion feature module on the NYU depth V2 dataset.

**Figure 13:** Experimental results of the upsampling optimization module on the NYU depth V2 dataset.

**Figure 14:** Comparative evaluation results of each algorithm on the NYU depth V2 dataset.

## Data Availability

The data used to support the findings of this study are available from the corresponding author upon request.
